# Anatomical Evaluation of Root and Root Canal Morphology of Permanent Mandibular Dentition among the Saudi Arabian Population: A Systematic Review

**DOI:** 10.1155/2022/2400314

**Published:** 2022-08-02

**Authors:** Mohammed Mashyakhy, Nada AlTuwaijri, Reuof Alessa, Nouf Alazzam, Bushra Alotaibi, Rahaf Almutairi, Riyad Alroomy, Gunaranjan Thota, Abdulaziz Abu Melha, Mazen F. Alkahtany, Khalid H. Almadi, Hitesh Chohan, Mohammed Tarrosh, Mubashir Baig Mirza

**Affiliations:** ^1^Restorative Dental Science Department, College of Dentistry, Jazan University, Jazan, Saudi Arabia; ^2^College of Dentistry, King Saud Bin Abdulaziz University for Health Sciences, Riyadh, Saudi Arabia; ^3^King Abdullah International Medical Research Center, Riyadh, Saudi Arabia; ^4^Restorative Dental Science Department, College of Dentistry, Majmaah University, Al Majmaah, Saudi Arabia; ^5^Restorative Dental Science Department, College of Dentistry, King Khalid University, Saudi Arabia; ^6^Restorative Dental Science Department, Division of Endodontics, College of Dentistry, King Saud University, Riyadh, Saudi Arabia; ^7^Conservative Dental Science Department, College of Dentistry, Prince Sattam Bin Abdulaziz University, Saudi Arabia

## Abstract

This study aimed to conduct a compendious review of root canal morphology of “permanent mandibular teeth in different regions of Saudi Arabia” to obtain a large sample representing the total population. A detailed search through the databases Web of Science, Scopus, and PubMed was conducted following the PRISMA guidelines. The data were analyzed based on the following inclusion criteria: original full-length original articles that reported the variables of interest “(number of roots, number of canals, Vertucci's classification system and C-shaped canals or mid-mesial canals)” of the mandibular teeth and conducted on Saudi subjects. The retrieved data were presented as frequencies and percentages. The results revealed that 56.6% of mandibular central incisors had one canal and Vertucci type I (56.6%), while 57.4% of the mandibular lateral incisors had one canal, with Vertucci types I and III most frequent. In mandibular canines, 91.8% had one canal and 8.2% had two canals. Most of the mandibular first premolars had one root (86.6%), while almost all mandibular second premolars (91.5%) had one canal, and 96.9% had Vertucci type I configuration. Among the mandibular first molars, three and four canals were prevalent in 58.7% and 40.6%, respectively. The majority of mesial roots had Vertucci type IV (60.6%), and most of distal roots had Vertucci type I (72.2%). Most of the mandibular second molars had three canals (87.3%) and showed Vertucci type IV (39.4%) canals for mesial roots and Vertucci type I (95.6%) for distal roots. The C-shaped canals were seen in 8% of first premolars and 9.8% of second molars. The middle mesial canal was found in 4.2% and 0.4% of first and second molars, respectively. This review could represent “the population of Saudi Arabia as the included samples were combined from different regions of the country.” Some variations were noticed within the same group of teeth from different regions. However, the overall results of combined samples were comparable to the other international studies.

## 1. Introduction

A successful root canal treatment (RCT) mainly depends on locating all root canals, debriding them entirely following the proper disinfection protocol and filling the root canal system (RCS) with an inert root filling material three dimensionally. [1] Daily, the wide range of RCSs poses a great challenge to clinicians in dental practice. Proper knowledge and the presence of advanced diagnostic tools to evaluate root canal anatomy are key to performing correct diagnoses and treatments and for achieving successful outcomes. The RCS involves obstacles, variations, and difficulties, especially posterior teeth, that negatively affect the main purpose of root canal treatment and reduce prognosis. [2, 3] Failure of RCT can be attributed to many factors; however, infection in missed, unfilled, or incompletely debrided canals is the main culprit. [4–9] Over the past decades, several studies have been carried out to investigate the external and internal anatomy of the root and root canal system, and these have found many variations. In addition, many techniques have been adopted to investigate the external and internal anatomy of teeth, such as “root sectioning, canal staining, tooth cleaning and microscopic examination” [10, 11], two-dimensional radiography [12, 13], and “three-dimensional (3D) technologies, including cone beam computed tomography (CBCT) [13] and microcomputed tomography (*μ*CT).” [14] Thus, the results of anatomical and morphological investigations may differ based on the study technique and the age, gender, and population of the group of interest. [15–17]

Several studies have been conducted utilizing various methodologies to evaluate mandibular “permanent dentition anatomy in various sub-populations in the Kingdom of Saudi Arabia (KSA) since 1999”. [3, 10, 13, 14, 18–33] Among some of those studies, the sample was defined as “Saudi population,” whereas in some others, it was described as “Saudi sub-population,” representing “different regions of Saudi Arabia, most of which were from the central region.” A critical concern is the representativeness of the samples to the whole Saudi population. A systematic review was found regarding the root and root canal variations of maxillary teeth among Saudi population. However, to the best of the authors' knowledge, there is no previous systematic review that has been conducted for mandibular teeth among Saudi population. [34]

Thus, the aim of this systematic review was to collect and combine all anatomical studies of mandibular permanent dentition conducted in the KSA to “achieve a large sample size that represents all regions of the country as a true KSA population sample.” The combined studies were then analyzed based on the number of roots, number of canals, and root canal configurations, and the findings were compared with those of other international studies.

## 2. Methodology

### 2.1. Research Question

This review was conducted following the guidelines of the “Preferred Reporting Items for Systematic Review and Meta-analysis (PRISMA).” The research question was “What is the prevalence of the number of roots, number of canals and root canal configuration of the permanent mandibular teeth among the Saudi population?”

### 2.2. Search Strategy

An online search through the main databases (Web of Science, Scopus, and PubMed) was conducted to retrieve the relevant studies by November 2021. Furthermore, a manual search was conducted on the hosting publishers (Wiley, ScienceDirect, and Springer) and individually on the well-known endodontic journals “(*Journal of Endodontics, International Journal of Endodontics, Australian Endodontic Journal, European Endodontic Journal and Saudi Endodontic Journal*)” to identify more related studies. Different combinations of the following words were used in the search strategy: “root canal morphology,” “root canal anatomy,” “root canal configuration,” “C-shaped canals,” “mid-mesial canals,” “mandibular teeth,” “mandibular,” “Kingdom of Saudi Arabia,” “Saudi Arabia,” “Saudi” and “KSA.”

Two authors (N.A. and R.A.) reviewed the extracted studies independently based on the following inclusion criteria: “original full-length articles that reported some or all of the study variables (number of roots, number of canals, Vertucci's classification system, C-shaped canals and mid-mesial canals) of the mandibular teeth, conducted on Saudi subjects (*in-vivo*) or teeth extracted from Saudi subjects (*in-vitro*), and published in English.” No time range was set for the search. All irrelevant studies, case reports and reviews, including abstracts, editorials, and studies with mixed populations, were excluded from the analysis. The initially extracted studies were firstly reviewed based on their titles and abstracts, and irrelevant studies were excluded. After that, the full text of the remaining studies was reviewed for eligibility. Moreover, the “reference lists of the studies that were included were screened for any possible relevant studies not included in the first evaluation.” In case of any disagreement between the two reviewers, a group discussion was opened with a third reviewer who was a specialist in endodontics (M.M.) to reach a consensus.

### 2.3. Data Extraction

The following parameters were extracted from the included studies: “authors (first author); year; region and city; research tool; investigated variables; number, gender, and age of the included subjects; type of teeth and number of teeth.” The main outcomes included the number of roots, the number of canals, and root canal morphology according to Vertucci's classification system. The secondary outcomes included the presence of C-shaped canals or mid-mesial canals. “The recruited information was extracted to a spread sheet file (MS Excel) and tabulated according to type of teeth. Frequency and percentage of each variable were reported, including the total of each category.”

## 3. Results

### 3.1. Study Selection

A total of 396 studies were retrieved from the search on the databases. In the first round of review, 45 studies were removed as duplicates, and 326 studies were excluded as irrelevant according to their titles and abstracts (e.g., abstracts, case report, editorials). In the second round of review, the full texts of the remaining 25 studies were reviewed for eligibility. Three studies were excluded because of the missing details on the main study variables. “Finally, 22 studies were included in the qualitative analysis (Figure 1).”

### 3.2. Characteristics of the Included Studies

*Main outcomes:* A total of 15 studies were conducted for the investigating of “number of roots, number of canals or root canal morphology.” Of them, 13 studies were performed on Saudi subjects (*in-vivo*), whereas two studies were performed on extracted teeth (*in-vitro*) of Saudi subjects. Regarding the method of investigation, 12 studies used CBCT, one study used panoramic X-ray (PA), while two studies used the drying method and dye (India ink) for the extracted teeth. Regarding the distribution of the studies, six studies were conducted in the central, six in the southern, two in the western, and one in the northern regions of the KSA. “A total of 4423 subjects were involved in these studies (three studies did not report the number of subjects).” It should be noted that two studies used the same subjects for the investigation of canine, first premolar, and second premolar teeth. Also, another three studies used the same subjects for the investigation of central, lateral, canine, first molar, and second molar teeth. The age of the subjects ranged from 13 years to 80 years (four studies did not report the age of the participants). Concerning gender distribution, 1909 were males, and 2102 were females (five studies did not report the gender distribution). The external and internal anatomy and morphology of 9868 mandibular teeth were investigated by these studies. Four studies investigated mandibular central and lateral incisors (*N* =1136 central and 1138 lateral incisors), three studies assessed mandibular canines (*N* =1558 teeth), five studies evaluated mandibular first and second premolars (*N* =1459 first premolars and 3495 second premolars), and four studies examined mandibular first and second molars (*N* =715 first molars and 367 second molars). It should be noted that some studies investigated more than one type of teeth (e.g., central and lateral incisors or first and second premolars or molars). With regard to the variables of interest, “13 studies reported the number of roots and canals and used Vertucci's classification system while two studies described the number of roots and canals. More details are presented in Table 1.”

*Secondary outcomes*: Seven studies investigated the C-shaped canals and mid-mesial canals of the mandibular first and second premolars and molars, with a total of 5070 teeth (*N* =3550 teeth for the C-shaped canals, and 1520 teeth for mid-mesial canals). All studies were conducted on Saudi subjects (*in-vivo*). Of these, five studies used CBCT and two studies used PA. There were 1328 subjects in these studies, with gender distribution of 634 males and 694 females, and the age ranged from 12 to 78 years (two studies did not report the number of subjects, gender distribution, or age of the participants). Regarding the distribution of the studies, five were conducted in the central region, one in the southern region, and one study was conducted on subjects from southern and western regions of the KSA. There were two studies that assessed the C-shaped canals of first and second premolars (*N* =673 first premolars and 637 second premolars) and four studies that assessed the C-shaped canals of first and second molars (*N* =926 first molars and 1421 second molars). There were three studies that assessed the C-shaped canals of more than one type of teeth in the same study. Also, there was one study that assessed the C-shaped canals of second molars in two regions of the KSA. Regarding the mid-mesial canals, one study assessed the mid-mesial canals of first and second molars, and another study assessed the mid-mesial canals of first molars only, with a total of 830 first molars and 690 second molars. More details are presented in Table 2.

### 3.3. Main Outcome Measures

#### 3.3.1. Mandibular Central Incisors

All four studies that investigated the mandibular central incisors reported one root for all teeth (*N* =1136 teeth [100%]) (Table 3). However, more than half of the teeth (*N* =643 teeth [56.6%]) had one canal and 43.4% (*N* =493 teeth) had two canals. “All studies reported Vertucci type I (56.6% of teeth), and Vertucci type III (38.2% of teeth).” However, one study reported Vertucci type II (1.7% of teeth) and Vertucci type IV (0.2% of teeth), and one study reported Vertucci type VII (0.9% of teeth), while two studies reported Vertucci type V (2.3% of teeth). No study reported Vertucci types VI and VIII.

#### 3.3.2. Mandibular Lateral Incisors

Four studies investigated the mandibular lateral incisors, with a total of 1138 teeth (Table 3). About 99.8% (*N* =1136 teeth) had one root, and only one study reported two teeth with two roots (0.2%). However, 57.4% (*N* =653 teeth) had one canal and 42.6% (*N* =485 teeth) had two canals. Regarding root canal morphology, all four studies reported Vertucci types I and III, with 57.4% (*N* =653) and 37.8% (*N* =430) of teeth, respectively. Vertucci type V was reported by three studies with 3.3% (*N* =37) of teeth, while one study reported Vertucci type II (*N* = 11 teeth [1.0%]), and another different study reported Vertucci type VII (*N* = 7 teeth [0.6%]). No study reported Vertucci types IV, VI, or VIII.

#### 3.3.3. Mandibular Canines

As shown in Table 3, three studies investigated the mandibular canines with a total of 1558 teeth, of which 97.9% (*N* = 1526 teeth) had one root and 2.1% (*N* = 32 teeth) had two roots. Most teeth had one canal (*N* = 1430 teeth [91.8%]) and 8.2% (*N* = 128 teeth) had two canals. In total, 92.7% (*N* = 1444 teeth) had Vertucci type I and 3.4% (*N* = 53 teeth) had Vertucci type III. Two studies reported Vertucci type V (*N* = 30 teeth), two studies reported Vertucci types II (*N* = 23 teeth) and IV (*N* = 6 teeth), while only one study reported Vertucci type VII (*N* = 2 teeth).

#### 3.3.4. Mandibular First Premolars

Four studies investigated the number of roots and number of canals of the mandibular first premolars (*N* =1459 teeth). Of these, 86.6% (*N* = 1263 teeth) had one root, 13.2% (*N* = 192 teeth) had two roots, and 0.2% (*N* = 4 teeth) had three roots. Regarding the number of canals, 75.3% (*N* = 1099 teeth) had one canal, 22.9% (*N* = 334 teeth) had two canals, and only 1.8% (*N* = 26 teeth) had three canals. The three studies that investigated the root canal morphology (*N* = 707 teeth) found Vertucci types I (79.3%), II (5.4%), III (4.7%), IV (2.1%), V (6.8%), and VI (0.4%. However, no study reported Vertucci type VII, only one study reported Vertucci type VIII (0.8%), and “one study reported other canal configurations (0.6%). More details are presented in Table 4.”

#### 3.3.5. Mandibular Second Premolars

Three studies investigated the number of roots and number of canals of 3495 mandibular second premolars. Mandibular second premolars with one root were the most prevalent (*N* = 3352 teeth [84.4%]), followed by mandibular second premolars with two roots (*N* = 141 teeth [4.0%]). Only one study reported mandibular second premolars with three roots (*N* = 2 teeth [0.1%]). Teeth with one canal were the most prevalent (*N* = 3199 teeth [91.5%]), followed by teeth with two canals (*N* = 290 teeth [8.3%]). Only one study reported teeth with three canals (*N* = 6 teeth [0.2%]), and no study reported teeth with four canals. Two studies investigated the root canal morphology of 2743 mandibular second premolars. All these studies reported Vertucci types I (96.9%), II (1.6%), III (0.1%), IV (0.8%), and V (0.3%). However, only one study reported Vertucci type VI (0.1%) and another study reported Vertucci type VIII (0.2%). More details are provided in Table 4.

#### 3.3.6. Mandibular First Molars

“Three studies investigated the number of roots and number of canals of mandibular first molars (*N* = 715 teeth).” Most teeth had two roots (*N* = 679 teeth [98.9%]), while 36 teeth (0.2%) had three roots. These studies also investigated the number of canals. More than half of the teeth (*N* = 420 teeth [58.7%]) had three canals, 270 (40.6%) teeth had four canals, and two studies reported five (0.7%) “teeth with two canals” (Table 5). “Only two studies investigated the root canal morphology of all roots” (*N* = 464 teeth). The most prevalent feature of the canal morphology of mesial roots was Vertucci type IV (60.6%), followed by Vertucci type II (33.8%). For distal roots, 72.2% (*N* = 335 teeth) had Vertucci type I, followed by Vertucci type III (*N* = 61 teeth [13.1%]). More details are presented in Table 6.

#### 3.3.7. Mandibular Second Molars

As shown in Table 5, only one study investigated the mandibular second molars (*N* = 338 teeth). Of these, two teeth (0.6%) had one root, 329 teeth (97.3%) had two roots, and seven teeth (2.1%) had three roots (Table 4). Most teeth (*N* = 295 teeth [87.3%]) had three canals, followed by two canals (*N* = 23 teeth [6.8%]) and 20 teeth (5.9%) had three canals. Regarding the Vertucci classification system, the most prevalent feature for mesial roots was Vertucci type IV (39.4%) followed by Vertucci type II (25.4%). However, the most prevalent feature was for the distal roots was Vertucci type I (95.6%) followed by Vertucci type V (2.6%). More details are shown in Table 6.

#### 3.3.8. Secondary Outcome Measures

*C-shaped canals*: Two studies explored the prevalence of C-shaped canals in mandibular first and second premolars (*N* =673 first premolars and 637 second premolars). The prevalence of C-shaped canals was 8% (*N* = 54 teeth) among first premolars and 3.5% (*N* = 22 teeth) among second premolars (Table 7). For mandibular first molars, two studies investigated C-shaped canals (*N* = 819 teeth). Of them, only one study found only one tooth (0.1%) with a C-shaped canal. For mandibular second molars, four studies (*N* = 1421 teeth) reported C-shaped canals in 139 teeth (9.8%). More details are given in Table 8.

*Mid-mesial canals*: Two studies (*N* = 830 teeth) investigated the mid-mesial canals in mandibular first molars and found 35 (4.2%) teeth with mid-mesial canals. However, only one study (*N* = 690 teeth) investigated the mid-mesial canals in mandibular second molars and found only three (0.4%) teeth with mid-mesial canals. More details are found in Table 9.

## 4. Discussion

Dentists may confront clinical challenges as a result of root canal morphology. One way in which the issues that may arise during endodontic therapy can be overcome is by “having knowledge of RCS in each group of teeth that allows potential difficulties during RCT to be addressed.” Nevertheless, it has been proven that numerous variables can contribute to RCS variations, such as age [35, 36], ethnicity [17, 37, 38], gender [38–41], and geographical area. [42] This disparity might be also attributed to differences in sample size, analytic technique, and statistical parameters used. In the following discussion, a variation in the population can be seen, which can be attributed to the above variables. This systematic review included all research on permanent mandibular teeth that matched the inclusion criteria in order to understand the RCS of Saudi permanent mandibular teeth.

### 4.1. Main Outcomes

#### 4.1.1. Mandibular Central Incisors

The present study reported higher second root canal prevalence (43.4%) when compared to other international studies. A systematic review pooled results from nine countries: Brazil, Belgium, China, Chile, Italy, Iran, Israel, Portugal, and Turkey. The pooled prevalence for the central incisors was 20.4% (15.0%–25.7%). This study was consistent with what was observed in Europe [36.8% (24.4%–49.3%)] and had a higher prevalence than in East Asia [7.6% (4.0%–11.3%)]. The systematic review findings, along with our findings, may speculate that the prevalence of the second canal in mandibular central incisor is higher when comparing non-Asians to Asians. [15] Our results found most studies reported Vertucci type I (56.6% of teeth) and Vertucci type III (38.2% of teeth). A study that was done in Iran found that Vertucci type I was prevalent in 72.7% of teeth, while Vertucci type III was prevalent in 4.7% of teeth. [43] In Malaysia, Vertucci type I and III were common in 94.9% and 1.0%, respectively. [44]

#### 4.1.2. Mandibular Lateral Incisors

This study also showed that the prevalence of second canal in mandibular lateral incisor was 42.6%, which was almost the same as our result with regard to the central incisor (43.4%). Martins et al. [45] also investigated the prevalence of the second canal in the mandibular lateral incisor. The pooled results from the aforementioned nine countries were 25.3% (20.0%–30.7%). Our results were consistent with the percentage in Europe also [37.5% (27.8%–47.2%)]. However, East Asia had less prevalence compared to ours and to Europe [17.2% (11.0%–23.4%)]. Consequently, we would also speculate that Asian had less second canal prevalence in mandibular lateral incisors compared to Saudi Arabia and Europe. [45]

Our results found most studies reported Vertucci type I (57.4% of teeth) and Vertucci type III (37.8% of teeth). In Iran, Vertucci I and III were prevalent in 70.6% and 3.7%, respectively. [43] In Malaysia, Vertucci type I and III were common in 87.8% and 3.8%, respectively. [44]

#### 4.1.3. Mandibular Canines

The present study showed the prevalence for second canal in mandibular canine was 8.2%. Martins et al. [45] investigated the prevalence of the second canal in the mandibular canines and found it was 5.9% (4.1%–7.7%) from the same aforementioned nine countries. This systematic review showed the prevalence for second mandibular canines in Europe was higher than those in the present study [9.8% (8.2%–11.5%)]. Moreover, second canals were lower in East Asian canine teeth [4.1% (2.8%–5.5%)]. [45]

Our findings revealed that the majority of studies reported Vertucci type I (92.7% of teeth) and Vertucci type III (3.4% of teeth). Vertucci I and III were common in Iran (71.8% and 2.8%, respectively). [43] In Turkey, Vertucci I and III were common in 87.8% and 9%, respectively. [46] In Malaysia, Vertucci type I was common in 95.1%; however, Vertucci III was not reported. [44]

#### 4.1.4. Mandibular First Premolars

The prevalence of two roots in mandibular first premolars was 13.2%, and the prevalence of two canals was 22.9% in our study. Vertucci I and V were the most common configuration (79.3% and 6.8%, respectively). In the Malaysian subpopulation, it has been shown that the prevalence of two canals was 18.7%. [44] The prevalence of two canals in the Spanish population was 20%. Vertucci canal configurations I and V were reported as the most common configurations in Malaysian, Spanish, and South Indian populations as well as ours. [44, 47, 48] Furthermore, the prevalence of two canals in Turkish population was approximately 25.5%. [49]

#### 4.1.5. Mandibular Second Premolars

The presence of the second canal in mandibular second premolars reported to be 4.0%, lower than in mandibular first premolars. This was consistent with the findings of a study done on the Spanish population 4.5%. [47] In the Malaysian subpopulation, the prevalence of two canals was lower than ours, at 0.5%. [44] In our study, Vertucci I was the most common configuration, followed by Vertucci II (96.9% and 1.6%, respectively). However, Vertucci I and V were the most common in the Spanish population, while Vertucci I and IV were the most common in the Malaysian population. [44, 47] Nevertheless, the prevalence in the Turkish population has been shown to be 29%. [49]

#### 4.1.6. Mandibular First Molars

The third root in mandibular first molar was prevalent in 5% of the studies pooled in this study. Four canals were prevalent in 40% and three canals were prevalent in 58.7%. In Belgium and Chile, the prevalence of three roots was 2.76% and 6.16%, respectively. [50] However, the prevalence of three roots in Asian countries was more than 30%. [11, 51] The mesial root of the mandibular first molar usually has two canals, Vertucci II and IV, according to a previous study that was consistent with this study. [11] Nevertheless, the most prevalent configurations in Belgium and Chili were Vertucci III and V. The distal root in this study has Vertucci I in 72.2%, which is consistent with the Chilean and Belgium populations. [50]

#### 4.1.7. Mandibular Second Molars

This study only found one study that investigated the root canal morphology of second mandibular molars. The prevalence of three roots was 2.1%, and the majority was two roots (97.3%). The majority had three canals 87.3%. In Belgium and Chile, the prevalence of three roots was 0.89% and 3.57%, respectively. Vertucci III and V were more prevalent in the mesial root in these populations, while Vertucci II and IV were more common in this study. The most common configuration of the distal root in all the above countries was Vertucci I. [50]

### 4.2. Secondary Outcome

#### 4.2.1. C-Shaped Canals in Mandibular Premolars

The prevalence of a C-shaped canal in mandibular first and second premolars was 8% and 3.5%, respectively. In Venezuela, the prevalence of a C-shaped canal in the mandibular first and second premolar was higher than in Saudi Arabia, as they were 28.94% and 7.14%, respectively. [52] Furthermore, it was higher in the USA (14%) for the first premolar. [53] However, it was much less in the Indian population for first and second mandibular premolar, which were 0.92% and 0.7%, respectively. [48]

#### 4.2.2. C-Shaped Canals in Mandibular Molars

The prevalence of C-shaped canals is higher in mandibular second molars than in mandibular first molars nine times in this systematic review (8% vs. 0.1%). Most studies were conducted in the mandibular second molar. The prevalence of C-shaped canals in the Emirates was higher than in Saudi Arabia (17.9%). It has been found that C-shaped canals are highly present in the Emirati population compared to Middle Eastern counties. [54] A previous research analyzed the racial predilection of C-shaped canals and found it was much more prevalent in Asians than in non-Asians. [55]

#### 4.2.3. Mid-Mesial Canals in Mandibular Molars

Few researches have been conducted in Saudi Arabia to assess mid-mesial canals prevalence in mandibular molars. The prevalence of the mid-mesial canal in the mandibular first molar was 4.2% in Saudi Arabia. Only one research investigated at the mandibular second molar and found that it has 0.4% prevalence mid-mesial canals. The prevalence of mid-mesial canals in mandibular molars in the Korean and Chinese populations were 0.35% and 2.7%, respectively. [50, 55] The previous research utilized CBCT to detect mid-mesial canals. In-vivo investigations, however, have revealed a higher prevalence of mid-mesial canals, as Azim et al. reported 46.2%. [56] Furthermore, Verisani et al. have reported greater prevalence of mid-mesial canals using micro-CT 18.6% for Brazilian and Turkish population. [57] This explained why different studies have wide variation in mid-mesial canals prevalence depending on methods used.

#### 4.2.4. Limitation and Further Recommendations

The 22 pieces of research from Saudi Arabia's various regions used a variety of methods and sample sizes and investigated different variables. As a result, demographics could not be gathered to assess the impact of gender and age on the current findings. Furthermore, because the number of investigations of different groups of teeth was minimal, the research was not split according to methodology or classified as in vivo or in vitro. Therefore, we just focused to address the main trait of anatomy, regardless of the variables.

Future multicenter research is recommended from all parts of the Kingdom of Saudi Arabia, and it should in vivo CBCT to enable the analysis of full dentition of sufficient patients to provide a large sample size that is representative of the whole Saudi population. Future studies should also gather more specific information on the influence of age and gender.

## 5. Conclusion

Despite the methodology, the anatomical studies presented in this study differ across various parts of the Kingdom of Saudi Arabia, even though they share the same ethnicity. The overall combined sample results fell within the range of other international studies. To increase the probability of successful endodontic therapy, root canal morphology must be thoroughly assessed. When periapical radiograph is unclear, a CBCT with a limited field of view would be used to comprehend the patient's tooth morphology to accomplish a favorable outcome.

## Figures and Tables

**Figure 1:** Flowchart of methodology according to PRISMA guidelines.

**Table 1:** Characteristics of the studies investigated number of roots, number of canals, and root canal morphology among Saudi population.

Study	Year	Region	Method	Investigation	No. subjects	Gender	Age	Type of teeth	No. teeth
Mohamed et al.	2021	Central	In-vivo; CBCT	#roots; #canals; Vertucci	94	62 M; 32 F	> 13	Centrals	188
								Laterals	188
Ghabbani et al.	2020	Western	In-vivo; CBCT	#roots; #canals; Vertucci	NR	NR	20 - 80	Centrals	498
								Laterals	498
Mashyakhy M.	2019	Southern	In-vivo; CBCT	#roots; #canals; Vertucci	208	100 M; 108 F	17 - 62	Centrals	410
								Laterals	412
Al-Fouzan et al.	2012	Central	In-vitro; dye	#roots; #canals; Vertucci	NR	NR	NR	Centrals	40
								Laterals	40
Almohaimede et al.	2021	Central	In-vivo; CBCT	#roots; #canals; Vertucci	1328	565 M; 763 F	18 - 74	Canines	694
Mashyakhy M.	2019	Southern	In-vivo; CBCT	#roots; #canals; Vertucci	208	100 M; 108 F	17 - 62	Canines	410
Al-Dahman et al.	2019	Central	In-vivo; CBCT	#roots; #canals; Vertucci	707	311 M; 396 F	16 - 79	Canines	454
Algarni et al.	2021	Southern	In-vivo; CBCT	#roots; #canals; Vertucci	166	NR	NR	First premolars	216
Chourasia et al.	2017	Southern	In-vitro; dye	#roots; #canals; Vertucci	NR	NR	NR	First premolars	100
Alam et al.	2020	Northern	In-vivo; CBCT	#roots; #canals	376	210 M; 166 F	15 - 60	First premolars	752
								Second premolars	752
Alfawaz et al.	2019	Central	In-vivo; CBCT	#roots; #canals; Vertucci	707	311 M; 396 F	16 - 79	First premolars	391
								Second premolars	343
Alghamdi & Khalil	2021	Western	In-vivo; CBCT	#roots; #canals; Vertucci	1200	600 M; 600 F	18 - 75	Second premolars	2400
Mashyakhy et al.	2019	Southern	In-vivo; CBCT	#roots; #canals; Vertucci	98	61 M; 37 F	15 - 50	First molars	174
Al-Nazhan S.	1999	Central	In-vivo; PA	#roots; #canals	246	NR	NR	First molars	251
Mashyakhy et al.	2021	Southern	In-vivo; CBCT	#roots; #canals; Vertucci	208	100 M; 108 F	17 - 62	First molars	290
								Second molars	367

**Table 2:** Characteristics of the studies investigated C-shaped and mid-mesial canals among Saudi population.

Study	Year	Region	Method	Investigation	No. subjects	Gender	Age	Type of teeth	No. teeth
Srivastava et al.	2019	Central	In-vivo; CBCT	C-shaped canals	156	82 M; 74 F	38.5	First premolars	276
								Second premolars	258
Mashyakhy et al.	2020	Southern	In-vivo; CBCT	C-shaped canals	208	100 M; 108 F	17 - 62	First premolars	397
								Second premolars	379
								First molars	290
								Second molars	367
Aldosimani et al.	2020	Central	In-vivo; CBCT	Mid-mesial canals	395	181 M; 214 F	31.5; 28.9	First molars	687
								Second molars	690
Alfawaz et al.	2019	Central	In-vivo; CBCT	C-shaped canals	487	228 M; 259 F	12 - 78	First molars	529
								Second molars	681
Srivastava et al.	2018	Central	In-vivo; CBCT	Mid-mesial canals	82	43 M; 39 F	13 - 70	First molars	143
Al-Fouzan K.	2002	Central	In-vivo; PA	C-shaped canals	NR	NR	NR	Second molars	151
Bahammam L	2018	Western	In-vivo; PA	C-shaped canals	NR	NR	NR	Second molars	168
		Southern	In-vivo; PA	C-shaped canals	NR	NR	NR	Second molars	54

**Table 3:** Number of roots, number of canals, and root canal configuration of mandibular incisors and canines among Saudi population.

Study (year)	Region City	Method	Sample	# roots (%)		# canals (%)		Vertucci's system (%)								
				1	2	1	2	I	II	III	IV	V	VI	VII	VIII	Others
Central incisors																
Mohamed et al. 2021	Center Qassim	CBCT In-vivo	188	188 (100.0)		77 (41.0)	111 (59.0)	77 (41.0)	19 (10.1)	86 (45.7)	2 (1.1)	5 (2.7)				
Ghabbani et al. 2020	Western Al-Madinah	CBCT In-vivo	498	498 (100.0)		236 (47.4)	262 (52.6)	236 (47.4)		228 (45.8)		24 (4.8)		10 (2.0)		
Mashyakhy M. 2019	Southern Jazan	CBCT In-vivo	410	410 (100.0)		302 (73.7)	108 (26.3)	302 (73.7)		108 (26.3)						
Al-Fouzan et al. 2012	Center Riyadh	Dye In-vitro	40	40 (100.0)		28 (70.0)	12 (30.0)	28 (70.0)		12 (30.0)						
Total			1136	1136 (100.0)		643 (56.6)	493 (43.4)	643 (56.6)	19 (1.7)	434 (38.2)	2 (0.2)	29 (2.3)		10 (0.9)		

Lateral incisors																
Mohamed et al. 2021	Center Qassim	CBCT In-vivo	188	188 (100.0)		90 (47.9)	98 (52.1)	90 (47.9)	11 (5.9)	83 (44.1)		4 (2.1)				
Ghabbani et al. 2020	Western Al-Madinah	CBCT In-vivo	498	498 (100.0)		250 (50.2)	248 (49.8)	250 (50.2)		212 (42.8)		29 (5.8)		7 (1.4)		
Mashyakhy M. 2019	Southern Jazan	CBCT In-vivo	412	410 (99.5)	2 (0.5)	285 (69.2)	127 (30.8)	285 (69.2)		123 (29.8)		4 (1.0)				
Al-Fouzan et al. 2012	Center Riyadh	Dye In-vitro	40	40 (100.0)		28 (70.0)	12 (30.0)	28 (70.0)		12 (30.0)						
Total			1138	1136 (99.8)	2 (0.2)	653 (57.4)	485 (42.6)	653 (57.4)	11 (1.0)	430 (37.8)		37 (3.3)		7 (0.6)		

Canines																
Almohaimede et al. 2021	Center Riyadh	CBCT In-vivo	694	674 (97.1)	20 (2.9)	625 (90.1)	69 (9.9)	639 (92.1)	11 (1.6)	20 (2.9)	5 (0.7)	17 (2.4)		2 (0.3)		
Mashyakhy M. 2019	Southern Jazan	CBCT In-vivo	410	399 (97.3)	11 (2.7)	372 (90.7)	38 (9.3)	372 (90.7)		25 (6.1)		13 (3.2)				
Al-Dahman et al. 2019	Center Riyadh	CBCT In-vivo	454	453 (99.8)	1 (0.2)	433 (95.4)	21 (4.6)	433 (95.4)	12 (2.6)	8 (1.8)	1 (0.2)					
Total			1558	1526 (97.9)	32 (2.1)	1430 (91.8)	128 (8.2)	1444 (92.7)	23 (1.5)	53 (3.4)	6 (0.4)	30 (1.9)		2 (0.1)		

**Table 4:** Number of roots, number of canals, and root canal configuration of mandibular first and second premolars among Saudi population.

Study (year)	Region City	Method	Sample	# roots (%)			# canals (%)				Vertucci's system (%)								
				1	2	3	1	2	3	4	I	II	III	IV	V	VI	VII	VIII	Others
First premolars																			
Algarni et al. (2021)	Southern Aseer	CBCT In-vivo	216	198 (91.7)	18 (8.3)		147 (68.1)	51 (23.6)	18 (8.3)		148 (68.5)	24 (11.1)	13 (6.0)	3 (1.4)	26 (12.1)	2 (0.9)			
Alam et al. (2020)	Northern Sakaka	CBCT In-vivo	752	608 (80.9)	144 (19.1)		536 (71.3)	216 (28.7)											
Alfawaz et al. (2019)	Center Riyadh	CBCT In-vivo	391	377 (96.4)	12 (3.1)	2 (0.5)	344 (88.0)	41 (10.5)	6 (1.5)		344 (88.0)	14 (3.6)	12 (3.1)	8 (2.0)	6 (1.5)	1 (0.3)		6 (1.5)	
Chourasia et al. (2017)	Southern Jazan	Dye In-vitro	100	80 (80.0)	18 (18.0)	2 (2.0)	72 (72.0)	26 (26.0)	2 (2.0)		69 (69.0)		8 (8.0)	4 (4.0)	16 (16.0)				4 (4.0)
Total			1459	1263 (86.6)	192 (13.2)	4 (0.2)	1099 (75.3)	334 (22.9)	26 (1.8)		561 (79.3)^*α*^	38 (5.4)^*α*^	33 (4.7)^*α*^	15 (2.1)^*α*^	48 (6.8)^*α*^	3 (0.4)^*α*^		6 (0.8)^*α*^	4 (0.6)^*α*^

Second premolars																			
Alghamdi & Khalil 2021	Western Jeddah	CBCT In-vivo	2400	2360 (98.3)	40 (1.7)		2350 (97.9)	50 (2.1)			2350 (97.9)	28 (1.2)	2 (0.1)	14 (0.6)	4 (0.2)	2 (0.1)			
Alam et al. (2020)	Northern Sakaka	CBCT In-vivo	752	664 (88.3)	88 (11.7)		540 (71.8)	212 (28.2)											
Alfawaz et al. (2019)	Center Riyadh	CBCT In-vivo	343	328 (95.6)	13 (3.8)	2 (0.6)	309 (90.1)	28 (8.2)	6 (1.7)		309 (90.1)	15 (4.4)	1 (0.3)	9 (2.6)	3 (0.9)			6 (1.7)	
Total			3495	3352 (95.9)	141 (4.0)	2 (0.1)	3199 (91.5)	290 (8.3)	6 (0.2)		2659 (96.9)^*β*^	43 (1.6)^*β*^	3 (0.1)^*β*^	23 (0.8)^*β*^	7 (0.3)^*β*^	2 (0.1)^*β*^		6 (0.2)^*β*^	

^*α*^The percentage is out of 707 teeth (the studies that investigated Vertucci system of 1^st^ premolars); ^*β*^ the percentage is out of 2743 teeth (the studies that investigated Vertucci system of 2^nd^ premolars).

**Table 5:** Number of roots and number of canals of mandibular first and second molars among Saudi population.

Study (year)	Region City	Method	Sample	# roots (%)				# canals (%)			
				1	2	3	4	1	2	3	4
First molars											
Mashyakhy et al. (2021)	Southern Jazan	CBCT In-vivo	290		274 (94.5)	16 (5.5)			2 (0.7)	187 (64.5)	101 (34.8)
Mashyakhy et al. (2019)	Southern Jazan	CBCT In-vivo	174		169 (97.1)	5 (2.9)			3 (1.7)	127 (73.0)	44 (25.3)
Al-Nazhan S. (1999)	Center Riyadh	PA In-vivo	251		236 (94.0)	15 (6.0)				106 (42.2)	145 (57.8)
Total			715		679 (95.0)	36 (5.0)			5 (0.7)	420 (58.7)	290 (40.6)

Second molars											
Mashyakhy et al. (2021)	Southern Jazan	CBCT In-vivo	338^*α*^	2 (0.6)	329 (97.3)	7 (2.1)			23 (6.8)	295 (87.3)	20 (5.9)
Total			338	2 (0.6)	329 (97.3)	7 (2.1)			23 (6.8)	295 (87.3)	20 (5.9)

*^*α*^* 29 C-shaped teeth were excluded from the total of 367.

**Table 6:** Root canal configuration of mandibular first and second molars among Saudi population.

Study (year)	Region City	Method	Sample	Type of root	Vertucci's system (%)								
					I	II	III	IV	V	VI	VII	VIII	Others
First molars													
Mashyakhy et al. (2021)	Southern Jazan	CBCT In-vivo	290	Mesial Roots	3 (1.0)	105 (36.2)	4 (1.4)	168 (57.9)	10 (3.4)				
				Distal Roots	200 (69.0)	9 (3.1)	50 (17.2)	2 (0.7)	29 (10.0)				
Mashyakhy et al. (2019)	Southern Jazan	CBCT In-vivo	174	Mesial Roots	3 (1.7)	52 (29.9)	3 (1.7)	113 (64.9)	2 (1.1)	1 (0.6)			
				Distal Roots	135 (77.0)	11 (6.3)	11 (6.3)	6 (3.5)	10 (5.8)	2 (1.2)			
Total			464	Mesial Roots	6 (1.3)	157 (33.8)	7 (1.5)	281 (60.6)	12 (2.6)	1 (0.2)			
				Distal Roots	335 (72.2)	20 (4.3)	61 (13.1)	8 (1.7)	39 (8.4)	2 (0.4)			

Second molars													
Mashyakhy et al. (2021)	Southern Jazan	CBCT In-vivo	338^*α*^	Mesial Roots	21 (6.2)	86 (25.4)	54 (16.0)	133 (39.4)	44 (13.0)				
				Distal Roots	323 (95.6)	3 (0.9)	3 (0.9)		9 (2.6)				
Total			338	Mesial Roots	21 (6.2)	86 (25.4)	54 (16.0)	133 (39.4)	44 (13.0)				
				Distal Roots	323 (95.6)	3 (0.9)	3 (0.9)		9 (2.6)				

^*α*^29 C-shaped teeth were excluded from the total of 367.

**Table 7:** Prevalence of C-shaped canals in mandibular premolars among Saudi population (%).

Study (year)	Region (City)	Method	Sample	C-shaped canals	
				Yes	No
First premolars					
Mashyakhy et al. (2020)	Southern Jazan	CBCT In-vivo	397	6 (1.5)	391 (98.5)
Srivastava et al. (2018)	Central Qassim	CBCT In-vivo	276	48 (17.4)	228 (82.6)
Total			673	54 (8.0)	619 (92.0)

Second premolars					
Mashyakhy et al. (2020)	Southern Jazan	CBCT In-vivo	379	3 (0.8)	376 (99.2)
Srivastava et al. (2018)	Central Qassim	CBCT In-vivo	258	19 (7.4)	239 (92.6)
Total			637	22 (3.5)	615 (96.5)

**Table 8:** Prevalence of C-shaped canals in mandibular molars among Saudi population (%).

Study (year)	Region (City)	Method	Sample	C-shaped canals	
				Yes	No
First molars					
Mashyakhy et al. (2020)	Southern Jazan	CBCT In-vivo	290	0 (0.0)	290 (100.0)
Alfawaz et al. (2019)	Central Riyadh	CBCT In-vivo	529	1 (0.2)	528 (99.8)
Total			819	1 (0.1)	818 (99.9)

Second molars					
Mashyakhy et al. (2020)	Southern Jazan	CBCT In-vivo	367	29 (7.9)	338 (92.1)
Alfawaz et al. (2019)	Central Riyadh	CBCT In-vivo	681	62 (9.1)	619 (90.9)
Bahammam L. (2018)	Western Jeddah	CBCT In-vivo	168	18 (10.7)	150 (89.3)
	Southern Albaha	CBCT In-vivo	54	14 (25.9)	40 (74.1)
Al-Fouzan K. (2002)	Central Riyadh	PA In-vivo	151	16 (10.6)	135 (89.4)
Total			1421	139 (9.8)	1282 (90.2)

**Table 9:** Prevalence of mid-mesial canals in mandibular molars among Saudi population (%).

Study (year)	Region (City)	Method	Sample	Mid-mesial canals	
				Yes	No
First molars					
Aldosimani et al. (2020)	Central Riyadh	CBCT In-vivo	687	9 (1.3)	678 (98.7)
Srivastava et al. (2018)	Center Qassim	CBCT In-vivo	143	26 (18.2)	117 (81.8)
Total			830	35 (4.2)	795 (95.8)

Second molars					
Aldosimani et al.(2020)	Central Riyadh	CBCT In-vivo	690	3 (0.4)	687 (99.6)
Total			690	3 (0.4)	687 (99.6)

## Data Availability

The data supporting the findings of this review are already included in this review.
